# Selenotranscriptomic Analyses Identify Signature Selenoproteins in Brain Regions in a Mouse Model of Parkinson’s Disease

**DOI:** 10.1371/journal.pone.0163372

**Published:** 2016-09-22

**Authors:** Xiong Zhang, Yang-Lie Ye, Hui Zhu, Sheng-Nan Sun, Jing Zheng, Hui-Hui Fan, Hong-Mei Wu, Song-Fang Chen, Wen-Hsing Cheng, Jian-Hong Zhu

**Affiliations:** 1 Department of Neurology, the Second Affiliated Hospital, Wenzhou Medical University, Wenzhou, Zhejiang, China; 2 Department of Preventive Medicine, Wenzhou Medical University, Wenzhou, Zhejiang, China; 3 Key Laboratory of Watershed Science and Health of Zhejiang Province, Wenzhou Medical University, Wenzhou, Zhejiang, China; 4 Institute of Nutrition and Diseases, Wenzhou Medical University, Wenzhou, Zhejiang, China; 5 Department of Food Science, Nutrition and Health Promotion, Mississippi State University, Mississippi State, Mississippi, United States of America; Consejo Superior de Investigaciones Cientificas, SPAIN

## Abstract

Genes of selenoproteome have been increasingly implicated in various aspects of neurobiology and neurological disorders, but remain largely elusive in Parkinson’s disease (PD). In this study, we investigated the selenotranscriptome (24 selenoproteins in total) in five brain regions (cerebellum, substantia nigra, cortex, pons and hippocampus) by real time qPCR in a two-phase manner using a mouse model of chronic PD. A wide range of changes in selenotranscriptome was observed in a manner depending on selenoproteins and brain regions. While *Selv* mRNA was not detectable and *Dio1& 3* mRNA levels were not affected, 1, 11 and 9 selenoproteins displayed patterns of increase only, decrease only, and mixed response, respectively, in these brain regions of PD mice. In particular, the mRNA expression of *Gpx1-4* showed only a decreased trend in the PD mouse brains. In substantia nigra, levels of 17 selenoprotein mRNAs were significantly decreased whereas no selenoprotein was up-regulated in the PD mice. In contrast, the majority of selenotranscriptome did not change and a few selenoprotein mRNAs that respond displayed a mixed pattern of up- and down-regulation in cerebellum, cortex, hippocampus, and/or pons of the PD mice. *Gpx4*, *Sep15*, *Selm*, *Sepw1*, *and Sepp1* mRNAs were most abundant across all these five brain regions. Our results showed differential responses of selenoproteins in various brain regions of the PD mouse model, providing critical selenotranscriptomic profiling for future functional investigation of individual selenoprotein in PD etiology.

## Introduction

Parkinson’s disease (PD), a major neurodegenerative disorder in elderly populations, is featured by progressive loss of dopaminergic neurons in substantia nigra. While a small portion of PD is hereditary, the majority of which is sporadic with a multifactorial etiology including oxidative stress, mitochondrial dysfunction, neuroinflammation and dysregulated protein degradation [1].

Selenium (Se), an essential trace element, exerts its biological functions mainly through selenoproteins that contain selenocysteine residues by decoding in-frame UGA codons with the help of a *cis*-acting selenocysteine insertion sequence at the 3’-untranslated region and a couple of *trans*-acting factors [2]. Human selenoproteome comprises 25 selenoproteins and includes the following families or groups [2]: 1) iodothyronine deiodinases (DIO), DIO1-3; 2) glutathione peroxidases (GPX), GPX1-4 and GPX6 (not present in mice); 3) thioredoxin reductases (TrxR), TrxR1, TrxR2 and TGR; 4) thioredoxin-like fold proteins in endoplasmic reticulum (ER), Sep15 and SelM; 5) SelW-like protein radixin (Rdx) family, SelH, SelT, SelW and SelV; 6) SelK and SelS that share similar topology; 7) others including SelI, SelP, SelO, SelN, methionine-*R*-sulfoxide reductase 1 (MsrB1, previously named as SelR and SelX) and selenophosphate synthetase-2 (SPS2). While Se deficiency in rats depletes more than 90% of Se in many organs, 71% of Se in the brain is retained [3]. This highlights a unique hierarchy of tissue Se retention under limited Se supply and suggests potentially critical roles of Se and selenoproteins in brain. This notion gains further supports from human studies as plasma Se status is positively associated with coordination and motor speed in elderlies [4].

Indeed, emerging evidence have linked Se and selenoproteins to PD. For instance, Se concentration and GPX activity are altered in plasma or erythrocytes of PD patients [5–7]. Similarly, while Se restriction or *Gpx1* knockout potentiates dopaminergic neurons to neurotoxins in mice, Se supplementation or *Gpx1* overexpression protects mice against the neuronal insults [8–15]. Although a couple of selenoproteins have been implicated in age-related brain degenerations [2,16], a lack of systematical analysis of all selenoproteins restricts a comprehensive understanding of Se-associated neurobiology in PD etiology. Herein, a prudent two-phase approach was applied to profile selenotranscriptome in five regions of brain in a mouse model of chronic PD.

## Materials and Methods

### Animals and chemicals

Male C57BL/6J mice (8–10 weeks old; 20–25 g; purchased from Experimental Animal Center of Wenzhou Medical University) were housed three to four animals per cage and given free access to pelleted chow diet and distilled water in an animal room maintained at constant temperature and humidity with a 12-h light-dark cycle. All animal experiments were approved by the Institutional Laboratory Animal Care and Use Committee at Wenzhou Medical University. 1-methyl-4-phenyl-1,2,3,6-tetrahydropyridine hydrochloride (MPTP-HCl; dissolved in saline) and probenecid (dissolved in basic Tris-HCl and diluted in saline) were purchased from Sigma (St. Louis, MI, USA).

### Treatments and sample collection

A chronic mouse model of PD was generated following the protocol as described previously [17,18]. Mice in the control group received saline as a vehicle, and mice in the PD group were intraperitoneally injected with MPTP-HCl (25 mg/kg) plus probenecid (250 mg/kg) (MPTPp) twice a week for 5 weeks (a total of 10 doses) before being sacrificed by cervical dislocation one week after the last injection. Five brain regions, including cerebellum, substantia nigra, cortex, pons and hippocampus, were collected and separated as instructed by procedures at http://www.mbl.org/anatomy_images/fresh/mbafr_1.html.

### RNA extraction and real-time qPCR

Brain samples were homogenized by using micro-pellet pestles, and total RNA was extracted (TriPure Isolation Reagent, Roche, Indianapolis, IN, USA) and reverse transcribed to cDNA (PrimeScript^TM^ RT reagent Kit, TaKaRa, Dalian, China) according to the manufacturers’ protocols. For real-time qPCR analyses, 50–100 ng of the cDNA was mixed with a 20 μl reaction system of FastStart Essential DNA Green Master (Roche, Indianapolis, IN, USA) and amplified in CFX96 Touch^TM^ real-time PCR detection system (Bio-Rad Laboratories, Hercules, CA, USA) with the cycling conditions as instructed by the manufacturer. Genes, encoded proteins, and primers were listed in Table 1.

**Table 1:** Primers used for quantitative real time PCR.

Gene	Protein	Primers
*Th*	Th	Forward: 5’-CAGCTGGAGGATGTGTCTCA-3’
		Reverse: 5’-GGCATGACGGATGTACTGTG-3’
*Dio1*	Dio1	Forward: 5’-CTGCCTGAGAGGCTCTACGT-3’
		Reverse: 5’-ACTTCATCTGGGAACACAGG-3’
*Dio2*	Dio2	Forward: 5’-GATCCTGCCAGTCTTTT-3’
		Reverse: 5’-ATTGGGAGCATCTTCAC-3’
*Dio3*	Dio3	Forward: 5’-GTCCTGGACACTATGGCCAA-3’
		Reverse: 5’-TCTTTGGAGCATTTGCACGT-3’
*Gpx1*	Gpx1	Forward: 5’-TGGACTGGTGGTGCTCG-3’
		Reverse: 5’-CGTCACTGGGTGTTGGC-3’
*Gpx2*	Gpx2	Forward: 5’-GGGCTGTGCTGATTGAGA-3’
		Reverse: 5’-CGGACATACTTGAGGCTGTT-3’
*Gpx3*	Gpx3	Forward: 5’-GGCTTCCCTTCCAACC-3’
		Reverse: 5’-AATTTCTGCTCTTTCTCCC-3’
*Gpx4*	Gpx4	Forward: 5’-ACGATGCCCACCCACT-3’
		Reverse: 5’-CCACGCAGCCGTTCTT-3’
*Txnrd1*	TrxR1	Forward: 5’-CCTATGTCGCCTTGGAATGTGC-3’
		Reverse: 5’-ATGGTCTCCTCGCTGTTTGTGG-3’
*Txnrd2*	TrxR2	Forward: 5’-GGCTCAGCGGCTCTTT-3’
		Reverse: 5’-CGCCACCGTGAACTCT-3’
*Txnrd3*	TGR	Forward: 5’-CAAGTTGATGACGGG-3’
		Reverse: 5’-TTGGCACAAGAGAGG-3’
*Sep15*	Sep15	Forward: 5’-CTGGCGACTGCGTTTC-3’
		Reverse: 5’-TCCTGACAGCACCCTCT-3’
*Selm*	SelM	Forward: 5’-TCGCCTAAAGGAGGTGAAG-3’
		Reverse: 5’-CATTTGGCTGAGTGGGATT-3’
*Selh*	SelH	Forward: 5’-GCCTATGGAGACGGTGGA-3’
		Reverse: 5’-GCGGTTTGGACGGGTT-3’
*Selt*	SelT	Forward: 5’-TTATCTCCCTCAACCAA-3’
		Reverse: 5’-CTCAGGAAGAAAACCAT-3’
*Sepw1*	SelW	Forward: 5’-TAAGCCCAAGTACCTCCA-3’
		Reverse: 5’-CCACATAGCCATCACCTC-3’
*Selv*	SelV	Forward: 5’-CAGGAGGAAGCATGCAAGA-3’
		Reverse: 5’-TGGTTTGGCAGCATTTCAG-3’
*Selk*	SelK	Forward: 5’-AAAGAAGAGGCTACGGG-3’
		Reverse: 5’-TTACCTTCCTCATCCACC-3’
*Sels*	SelS	Forward: 5’-CTTTGCGAGGAGGTGGTTAT-3’
		Reverse: 5’-CCTTGCTAATGTCAGAGCGA-3’
*Seli*	SelI	Forward: 5’-TCCGTGTTTGCTCTTCA-3’
		Reverse: 5’-CGTGCTGCTCATTTGG-3’
*Sepp1*	SelP	Forward: 5’-GGCCGTCTTGTGTATCACCT-3’
		Reverse: 5’-TGGTGTTTGTGGTGGCTATG-3’
*Selo*	SelO	Forward: 5’-CCAGCGTGGGACGAGAT-3’
		Reverse: 5’-CTGCCATTCAGCAACCAT-3’
*Msrb1*	MsrB1	Forward: 5’-CTTCGGAGGCGAGGTT-3’
		Reverse: 5’-TGGGTGGATGGTTTCAG-3’
*Sepn1*	SelN	Forward: 5’-GACTTCCCCTTCTGGTT-3’
		Reverse: 5’-TGTTGCTGGTCTCACTG-3’
*Sephs2*	SPS2	Forward: 5’-GTGCCGTGGTAGGAGATGTG-3’
		Reverse: 5’-GCAGTCCTGTTTAGAGTAGCCATA-3’
*Actb*	β-actin	Forward: 5’-CTGTCCCTGTATGCCTCTG-3’
		Reverse: 5’-ATGTCACGCACGATTTCC-3’

### Data presentation and analyses

Two sets of control and PD mice were generated sequentially to represent the discovery phase and replication phase, respectively. The qPCR analyses were performed for the discovery (n = 4, except for substantia nigra) and replication (n = 3) phases. The mRNA expression was first calculated and presented as a comparative cycle threshold value (2^ (-ΔΔC_T_)), followed by normalization to the mean of the control group. Two-tailed Student’s *t*-test was used to determine differences between the control and PD groups. Data were expressed as means ± SE. Statistical difference was set as *p* < 0.05. A trend of difference was considered when the change between the control and PD groups exceeded 10%. Statistical analysis as a whole (two phases combined, n = 7) was performed only when a repeatability was detected, that is, either statistical difference or a trend is present at both discovery and replication phases, and meanwhile the change (increase or decrease) is in the same direction. As sample volume in some sub-brain regions of mice was small and results from similar studies were not always consistent due to either subtle difference or large variations, this two-phase approach was used for qPCR analyses to boost confidence and improve accuracy.

The heat map was made by Heatmap Illustrator version 1.0 (HemI, version 1.0) for windows. Volcano plots were drawn with fold change (log2) as X-axis and p value (-log10) as Y-axis. The abundance of selenoprotein mRNA was normalized with that of β-actin, which was calculated based on the equation below,

$$Exp(g,r)=\frac{2^{-\Delta {CT}_{g,r}}}{2^{-\Delta {CT}_{\beta ,r}}}$$

where “*Exp*”, “g”, “r”, and “β” denotes mRNA expression, a selenoprotein gene, a certain brain region, and β-actin gene.

### Immunohistochemistry

Mice were euthanized and perfused via the left ventricle with saline and 4% paraformaldehyde sequentially. Brains were removed, fixed overnight in 4% paraformaldehyde before being dehydrated in ethanol, and processed using standard procedures for paraffin-embedded samples. The antibody against Gpx1 was from Abcam (Cambridge, MA, USA) and Gpx4 was from was from Santa Cruz Biotechnology (Santa Cruz, CA, USA). Immunohistochemistry was performed by using a kit from ZSGB-BIO Co. (Beijing, China) according to the manufacturer’s instructions.

## Results

### The selenotranscriptome is widely altered in the PD mice

As described in materials and methods, statistical analyses in the combined group (named total) were considered only when repeatability was evidenced in the discovery and replication phases. Following the MPTPp administrations, the mRNA expression of tyrosine hydroxylase (TH, a marker of dopaminergic neuron) in substantia nigra was dramatically decreased (42.5 and 68.2% in the discovery and replication phase, respectively; 55.4%, total) (Fig 1), validating the model of PD in mice.

**Fig 1:** The mRNA expression of tyrosine hydroxylase (*Th*) in substantia nigra. *, *p* < 0.05, compared to control.

The mRNA levels of Dio family were not changed in the PD mice except a trend of *Dio2* decrease in the pons region (Fig 2A). In contrast, there was a general declining pattern of the Gpx family in the PD mice, particularly in the region of substantia nigra (Fig 2B). In particular, the mRNA level of *Gpx1* declined by 20.6% and 21.1% (p < 0.05) in substantia nigra and hippocampus of the PD mice, respectively. The mRNA level of *Gpx2* was reduced by 17.2%, 21.8% (p < 0.05) and 21.4% (p = 0.17) in cerebellum, hippocampus and substantial nigra, respectively. The mRNA level of *Gpx3* was reduced by 43.5%, 39.8% (p < 0.05), 18.8% (p = 0.11) and 19.5% (p = 0.083) in cerebellum, substantial nigra, cortex and hippocampus, respectively. The *Gpx4* mRNA was down-regulated (28.2%, p < 0.05) in the substantial nigra. As a note, there was a significant decrease (p = 0.02) for the *Gpx4* mRNA in the hippocampus of the total (two phases combined) group, although this region failed the repeatability test as described in the methods section.

**Fig 2:** Two-phase mapping of selenotranscriptome in the cerebellum, substantia nigra, cortex, pons and hippocampus of control and PD mice. The selenotranscriptome is categorized as iodothyronine deiodinases (A), glutathione peroxidases (B), thioredoxin reductases (C), thioredoxin-like endoplasmic reticulum proteins (D), the Rdx family members (E), SelK and SelS (F), and others (G). The black and white bars indicate those with repeatability in the discovery and replication phases. *, p < 0.05, compared to control. ^#^, ^##^, and ^###^ indicates a trend of difference with percentage of change at 10–15%, 15–20%, and > 20% respectively. The left and right bars for each of the sub-brain regions denote control and PD mice, respectively.

In the TrxR family (Fig 2C), their mRNA transcripts can be up- or down-regulated in different regions of the PD mouse brain. The mRNA level of *Txnrd1* was decreased by 30% and 16.3% (p < 0.05) in substantial nigra and pons, respectively, but elevated by 16.9% (p < 0.05) in cortex of the PD mice. *Txnrd2* mRNA was also decreased (24.2%, p < 0.05) in the substantial nigra, but increased in the cortex and the pons by 36.7% and 24.6% (p < 0.05), respectively. The mRNA level of *Txnrd3* was decreased only in hippocampus (21.9%, p < 0.05).

The mRNA level of *Sep15* was reduced by 28.2% and 18.0% (p < 0.05) in substantia nigra and hippocampus of the PD mice, respectively (Fig 2D). In contrast, the expression of SelM was elevated by 21.6% (p < 0.05) in the cerebellum, but decreased by 15.3% and 25.9% (p < 0.05) in the substantia nigra and the cortex, respectively.

Strikingly, the Rdx family of selenoproteins exhibited a consistent trend of decreased mRNA expression in substantia nigra but increased expression in some other regions of the PD mouse brain (Fig 2E). The mRNA levels of *Selh*, *Selt*, *Sepw1*, *Selk* and *Sels* were decreased by 31.3, 11.6, 40, 23.4, and 31.5% (p < 0.05) in the substantia nigra, respectively. In contrast, the mRNA level of *Selh* was increased by 22.8% (p = 0.062) and 16.2% (p < 0.05) in the cerebellum and the pons, respectively, and that of *Selt* displayed an increasing trend by 17% (p = 0.1) and 21.8% (p = 0.065) in cortex and pons, respectively. Similarly, the mRNA levels of *Sepw1* were increased by 21.8% (p = 0.06), 20.5% and 29.3% (p < 0.05) in cerebellum, cortex and hippocampus, respectively. *Selv* mRNA was not detectable in any of the five brain regions, which was likely attributed to its testis-specific distribution [19]. The mRNA level of *Sels* was also decreased (14.5%, p = 0.16) in hippocampus of the PD mice (Fig 2F).

For the rest of selenoproteins (Fig 2G), the mRNA level of *Seli* was decreased by 15%, 21.1%, and 16.3% (p < 0.05) in substantia nigra, cortex, and hippocampus, respectively, and that of *Sepp1* was decreased by 15.6% and 16.7% (p < 0.05) in substantia nigra and pons of the PD mice, respectively. Besides, there was a declining pattern of *Sepp1* expression in all the five brain regions and as a note, a statistical difference was present in the cerebellum (p = 0.01) and cortex (p = 0.04) of the total group, although the designed repeatability was not detected. *Selo* mRNA level was decreased by 20.8% (p < 0.05) in substantia nigra, but increased by 29% and 19.4% (p < 0.05) in cerebellum and pons of the PD mice, respectively. The mRNA level of *Msrb1* was decreased by 19.1% and 12.1% (p < 0.05) in substantia nigra and cortex, respectively, but increased by 19.2% (p < 0.05) in hippocampus of the PD mice. The *Sepn1* mRNA level was increased by 33.2% (p < 0.05) in the cerebellum, but decreased by 15.5% (p < 0.05) in the pons. The mRNA level of *Sephs2* was increased by 12.7% and 18.4% (p < 0.05) in cerebellum and cortex of the PD mice, respectively.

### Selenotranscriptome is distinct in different brain regions of PD mice

The volcano plots showed up-regulated and down-regulated selenoprotein mRNAs and the genes with significant changes (Fig 3A), and the heat map displayed the extent of changes (Fig 3B). These results suggest a distinct pattern of selenotranscriptome in various regions of the PD mouse brain. Except *Dio1-3*, *Sepn1*, *Sephs2*, *and Txnrd3*, the mRNA expression of the other 17 selenoproteins concordantly declined in substantia nigra of the PD mice (Fig 3B and 3C). In contrast, while the majority of selenotranscriptome remained unchanged in the other four brain regions of PD mice, up- and down-regulation of selenoproteins both existed in these brain areas (Fig 3A and 3C). In the cortex, while the mRNA levels of *Sephs2*, *Sepw1*, *Txnrd1-2* and *Selt* were increased, those of *MsrB1*, *Seli*, *Selm*, and *Gpx3* were decreased. In the hippocampus, the mRNA levels of *MsrB1* and *Sepw1* were increased, whereas those of *Gpx1-3*, *Seli*, *Sep15*, and *Sels* were decreased (Fig 3C; left panel). In the cerebellum, while the mRNA levels of *Selm*, *Selo*, *Sephs2*, *Sepn1*, *Selh*, and *Sepw1* were increased, those of *Gpx2-3* were decreased. In the pons region, the mRNA levels of *Selh*, *Selo*, *Txnrd2*, and *Selt* were increased, whereas those of *Sepn1*, *Sepp1*, *Txnrd1*, and *Dio2* were dropped (Fig 3C; right panel).

**Fig 3:** The changes of selenotranscriptome in the five brain regions of PD mice. (A) Volcano plots showing up-regulated (X axis > 0) or down-regulated (X axis < 0) selenoprotein mRNAs. Labeled are genes with significant difference (*p* < 0.05; above the X axis) or with a trend of difference (changes > 10%; underlined). *d2*, *Dio2; g1*, *Gpx1; g2*, *Gpx2; g3*, *Gpx3; g4*, *Gpx4; t1*, *Txnrd1; t2*, *Txnrd2; t3*, *Txnrd3; 15*, *Sep15; m*, *Selm; h*, *Selh; t*, *Selt; w*, *Sepw1; k*, *Selk; s*, *Sels; i*, *Seli; p*, *Sepp1; o*, *Selo; r*, *MsrB1; n*, *Sepn1; s2*, *Sephs2*. (B) A heat map displaying the extent of changes. The color scale ranges from saturated red (0.327) to white (-0.034) to saturated blue (-0.435). Red and blue colors represent increased and decreased expression, respectively. (C) A brain diagram illustrating the responses in each brain region. Saturated red and blue colors represent increased and decreased expression (p < 0.05), respectively. Pale colors represent a trend of difference (> 10%). Each of the brain regions is labeled symmetrically.

### The relative abundance of selenoprotein mRNAs in the brain regions

The mRNA levels of five selenoproteins (*Gpx4*, *Sep15*, *Selm*, *Sepw1* and *Sepp1*) were most abundant, followed by *Gpx1*, *Selt* and *Selk*, in all the five brain regions. In contrast, in addition to the undetectable *Selv*, five genes (*Dio1*, *Dio3*, *Gpx2*, *Txnrd2*, and *Txnrd3*) were barely detectable in any of the brain regions, and four genes (*Sels*, *Selo*, *MsrB1* and *Sephs2*) were detected at a low level (Fig 4). Furthermore, *Dio2* was barely detectable in the substantial nigra but expressed at a medium level in other four brain areas. *Gpx3* was detectable only in substantial nigra and pons of the PD mice. *Txnrd1* and *Seli* were modestly expressed only in the pons and the hippocampus, respectively, and at a low level in other areas of the PD mouse brain. *Selh* was expressed highly in the cerebellum, modestly in the substantial nigra and the pons, and at a low level in the cortex and the hippocampus. *Sepn1* was expressed at a low level in the cerebellum and the substantial nigra, but was barely detectable in other brain regions (Fig 4).

**Fig 4:** Relative abundance of selenotranscriptome in the brain regions of control mice. The individual mRNA expression level was calculated and normalized with their respective β-actin expression in the brain region. The relative abundance of selenoprotein mRNA expression was divided into the four groups: barely detectable (values < 0.1), low expression (0.1–0.5), medium expression (0.5–1), and high expression (> 1).

### Analysis of Gpx1 and Gpx4 protein expression in three brain regions of control and PD mice

In order to understand whether the mRNA changes are in accordance with the changes in protein levels, two selenoproteins, Gpx1 and Gpx4, were assessed by immunohistochemistry in the substantia nigra, cortex and hippocampus of control and PD mice. As expected, the substantia nigra of PD mice exhibited a dramatic reduction in TH levels compared with the control sections. Similar to the changes in mRNA levels, the positive staining of Gpx1 and Gpx4 was obviously reduced in the substantia nigra of PD mice, but remained unchanged in the cortex (Fig 5). The level of Gpx1 was apparently reduced in the hippocampus of PD mice. Interestingly, the density of Gpx4 staining also appeared decreased in the hippocampus (Fig 5), where its mRNA level showed a reduction in the total group as noted earlier. Overall, these results suggest similar responses of Gpx1 and Gpx4 between protein and mRNA levels in the three brain regions of PD mice.

**Fig 5:** Gpx1 and Gpx4 protein expression in the substantia nigra, cortex and hippocampus of control and PD mice determined by immunohistochemistry. Representative images were presented following visual inspections of the brain slices from three control and PD mice, respectively. Bar size, 20 μM. TH, tyrosine hydroxylase. Arrows indicate examples of positive staining in brown. Blue color indicates nuclei.

## Discussion

Body Se status has been linked to PD in animal [8,10–12] and humans [4,5] studies. Nonetheless, it remains largely elusive whether Se-containing proteins are implicative in this disease. The current study is the first to systematically analyze selenotranscriptome in a mouse model of chronic PD in five areas of the brain.

Zhang et al [20] previously analyzed the expression pattern of selenotranscriptome in the brain by extracting data from genome-wide Atlas of gene expression in the adult mouse brain [21]. They identified six abundant selenoproteins in the brain (SelM, SelP, SelK, Sep15, SelW and Gpx4) and five selenoproteins that express at undetectable to lowest levels (Dio1, Dio3, SelV, TrxR2 and Gpx2). Our results are comparable to the Atlas dataset based on normal brain except for SelK, which expresses highly in two regions (cerebellum and pons) and modestly in the remaining three. Furthermore, in addition to the above five minutely expressed selenoproteins, we found TrxR3 expression to be low in the brain of PD mice. A microarray dataset examining gene expression in MPTP-treated mouse brains have been previously reported [22]. Although providing near genome wide coverage, one disadvantage of many of them is the lack of statistical power to identify relatively small changes. In contrast, the major advantage of the current targeted approach is that we likely obtain enough power to observe small changes, and the use of discovery and replication phases suggests that they are likely to be true differences.

The main physiological function of GPX is to catalyze the glutathione-dependent removal of hydrogen peroxide. While mice deficient in *Gpx1* are more susceptible to MPTP-induced dopaminergic cell death, *Gpx1*-overexpressing mice display increased resistance to 6-hydroxydopamine neurotoxicity in substantia nigra [13–15]. In accordance, we found that Gpx1 mRNA expression is significantly reduced in the substantia nigra of PD mice. These results suggest that Gpx1 may alleviate the vulnerability to loss of dopaminergic neurons in PD mice [16]. Interestingly, it has also been reported that GPX1 activity in substantia nigra decreases with age in humans [23]. A neuronal role of Gpx2, also known as gastrointestinal Gpx, is less prominent due to its low expression in brain; however, its expression is reduced in several regions of the PD mouse brain. It remains to be determined such reduction of *Gpx2* expression is a cause or consequence of PD. The expression of *Gpx3*, also known as extracellular or plasma Gpx, is also reduced in the substantia nigra of PD mice, which is in line with previous reports as determined in erythrocytes of PD patients [6,7]. Knockout of *Gpx4*, also known as phospholipid hydroperoxide Gpx, in mice results in embryonic lethality, suggesting the essentiality of this selenoprotein [24]. Together with our result demonstrating reduction of *Gpx4* mRNA expression specifically in substantia nigra of the PD mice, the observations that dopamine quinone can covalently modify and decrease the expression of mitochondrial Gpx4 in rats [25] suggest that Gpx4 may protect dopaminergic neurons in PD. Taken together, it appears that the whole GPX family or total GPX activity play critical roles in the susceptibility to PD risk.

In contrast to Gpx family, the *Dio1-3* mRNA levels are not significantly affected in the brain regions of PD mice. Although hypothyroidism and abnormal thyroid hormone levels are sometimes reported in PD patients [26,27], our results suggest little or no role of Dios in the PD brain. This is indeed not surprising, considering the nature of Dio family members in catalyzing deiodination of thyroid hormone and their relatively low abundance in the brain. The TrxRs are members of the oxidoreductase family and reduce protein disulfide bonds by using thioredoxin as a reducing agent. While TrxR1 (mainly localized in cytosolic) is modestly expressed, TrxR2 (mainly localized in mitochondria) and TrxR3 (primarily expressed in testis) are barely detectable in the five brain regions in the PD mice. The observation that *Txnrd1* expression is decreased in the substantia nigra of PD mice is in line with a recent report demonstrating reduced expression of TrxR1 mRNA and protein in substantia nigra of PD mice induced by MPTP [28]. Furthermore, nervous system-specific knockout of *Txnrd1* in mice leads to smaller body size with ataxia and tremor while mice deficient in *Txnrd2* develop normally [29]. These studies indicate that TrxR1 underexpression may be positively associate with the pathogenesis of PD.

A role of Sep15, SelM, SelK, and SelS in PD has not been reported. Sep15 and SelM have been implicated in protein folding by catalyzing the reduction or rearrangement of disulfide bonds in ER or secretory proteins [30]. Although SelM is known to regulate the pathogenesis of Alzheimer’s disease through activation of ERK and inhibition of β/γ-secretase and Tau phosphorylation [31], knockout of *Selm* does not lead to cognitive deficits in mice despite of the obesity phenotype [32]. In addition to being linked to inflammation and immune responses [2], SelK and SelS have been implicated in ER-associated degradation of misfolded proteins [33,34]. Interestingly, a large body of evidence suggests ER stress as an early event of PD pathogenesis [35]. Altogether, it is of future interest to investigate the pathogenesis of PD in the context of ER-associated function, substantia nigra-specific expression, and changes of ER selenoproteins in PD mice.

Of the selenoproteins in the Rdx family, SelV expression is restricted in testes [19] and is not detectable in the brain of PD mice. In contrast, the mRNA expression of SelW overall is the most abundant in the mouse brain. Of note, the expression of SelW in the brain of rats and sheep is highly persevered under Se deficiency, even to the extent with dietary Se deprivation for two generations [36,37]. Although the exact function awaits further investigation, such robust retention indicates a critical role of SelW in the brain. Consistent with this notion, *Sepw1* mRNA level in substantia nigra drops the greatest among selenotranscriptome in the PD mice. Interestingly, *Sepw1* mRNA is slightly up-regulated in cerebellum, cortex and hippocampus in the PD mice, which is in line with a report showing increased SelW expression in the cortex of PD patients [38]. Because SelW is downregulated in SH-SY5Y neuroblastoma cells after glutathione depletion by methylmercury treatment [39] and siRNA knockdown of SelW inhibits cell cycle progression and epithelial cell proliferation [40], SelW may regulate cell survival in the PD brain. Furthermore, the other two Rdx family members, *Selh* and *Selt*, display a similar pattern of mRNA expression as that of *Sepw1*. While SelH has been implicated in maintaining genomic stability and redox regulation [41] and SelT is identified as a target of the pituitary adenylate cyclase-activating polypeptide regulating Ca^2+^ levels [42], exact roles of these two selenoproteins in PD brain await further investigation.

SelP is considered as a main transporter carrying Se to peripheral tissues, in particular, brain and testis. Knockout of *Sepp1* in mice leads to very low concentration of Se in brain and severe neurological problems such as poor motor coordination [43,44]. In line with the current study, SelP expression is significantly decreased in substantia nigra of PD subjects [45]. Furthermore, *Sepp1* mRNA level appears decreased in the other four brain regions in PD mice. The mRNA levels of *Seli*, *Selo* and *Msrb1* are also reduced in substantia nigra of the PD mice. Although little is known about the function of SelI and SelO, MsrB1 has been shown to repair oxidized methionine residues on proteins [2].

Since substantia nigra is the primary site of action for MPTP, the changes in selenotranscriptome may reflect specific responses of dopaminergic neurons to oxidative stress and mitochondrial dysfunction that subsequently lead to cell death. Alternatively, they could also be general events that occur during cell death that may not be specific to dopaminergic neurons or particularly relevant to PD. The validation results show that the protein expression changes of Gpx1 and Gpx4 evaluated by immunohistochemistry are in line with their changes in mRNA levels in response to the induction of PD mouse model. However, in substantia nigra it is likely that the decrease of these selenoproteins is simply due to the loss of neurons instead of a true intracellular response, particularly when the protein is predominantly neuronal expressed. Thus, it remains to be further investigated for individual selenoproteins to understand its cause-effect relationship with PD and its distribution and actual intraneuronal expression in substantia nigra of PD.

In summary, the results presented herein have demonstrated a wide range of changes in the selenotranscriptome of PD mice, accompanied with a unique signature of differential expression for each selenoprotein gene in the brain regions. Of note, most of the genes are down-regulated in the substantia nigra of PD mice, suggesting that selenoproteins may play a key role in the protection against PD risk. It remains to be further clarified whether these alterations contribute to the pathogenesis or simply the consequence of PD.
